# Thoracic endovascular aortic repair for type B aortic dissection after renal transplantation

**DOI:** 10.18632/oncotarget.21399

**Published:** 2017-09-30

**Authors:** Chang Shu, QingGen Xiong, Jian Qiu, MingYao Luo, Kun Fang

**Affiliations:** ^1^ Department of Vascular Surgery, The Second Xiangya Hospital of Central South University, Changsha, 410011, China; ^2^ Center of Vascular Surgery, Fuwai Hospital, National Center for Cardiovascular Diseases, Chinese Academy of Medical Sciences and Peking Union Medical College, Beijing, 100037, China

**Keywords:** type B, aortic dissection, TEVAR, renal transplantation, follow up

## Abstract

Thoracic endovascular repair (TEVAR) is an effective treatment for type B aortic dissection (TBAD). Here, we evaluated the early-midterm effectiveness and safety of TEVAR for treating TBAD patients after renal transplantation. Six patients with TBAD treated with TEVAR after renal transplantation were recruited between February 2012 and December 2016. They were then followed up with clinical examinations and computed tomography angiography (CTA). TEVAR was successfully performed in all patients (100%), and the primary tear sites were well covered by stents with or without coverage of the left subclavian artery. No severe complications occurred in any patient during perioperative period. The one-year survival rate was 100%, one patient died of renal graft failure and heart failure four years after TEVAR; the remaining five patients (83.3%) survived and exhibited no severe complications. Our findings show that TEVAR provides satisfactory short-midterm results for TBAD patients after renal transplantation. Moreover, our experience shows that it need relative longer proximal landing zone to prevent the endoleak and recurrence. However, regular hematodialysis, long-term immunosuppressive therapy, and blood pressure control remain crucial factors to prolong survival. Long-term follow-up studies are needed to evaluate the long-term prognosis in these patients.

## INTRODUCTION

Aortic dissection (AD) is a catastrophic cardiovascular disease, with a prevalence of 10/100,000 in elderly adults [1]. Among aortic dissections (ADs), 30% are type B aortic dissections (TBADs). The mortality rate in TBADs is approximately 10% [2, 3]. AD is often associated with hypertension, atherosclerosis, and genetic tunica media degeneration, such as in Marfan’s syndrome. However, TBADs after renal transplantation are rarely reported. These patients tend to have hypertension, weak vessels, and vascular calcification (VC), which worsens with time [4]. VC may cause stenosis and even occlusion of the renal artery, resulting in renal hypertension and graft failure. The reported incidence of hypertension following successful renal transplantation varies from 13 to 80% [5-9]. In addition, accumulated excess volume and transplant kidney dysfunction contribute to hypertension. The unstable blood pressure (BP) and atherosclerotic aorta make the rupture of AD after renal transplantation unpredictable.

Thoracic endovascular repair (TEVAR) is an effective and minimally invasive treatment compared to open surgery, and is currently widely adopted in treating TBADs. The ultimate goals of TEVAR for TBADs are to cover the entry and re-entry tear site of the dissection and restore normal blood flow in the true lumen [2, 10-11]. TEVAR leads to the collapse of the false lumen and results in partial or complete thrombosis of the false lumen [12]. However, TBADs after renal transplantation are prone to rupture and are vulnerable to damage caused by renal dysfunction, and thus, the positioning of the proximal landing zone and the protection of renal function are critical for this type of TBAD. Reports about TEVAR treatment of patients with TBAD after renal transplantation are rare. Here, we report six TEVAR cases to treat patients with TBAD after renal transplantation. Based on our experience, we have summarized the treatment process, prognosis, and short-midterm follow-up outcomes.

## RESULTS

TEVAR was successfully performed in all patients, including the coverage of the primary tear site with or without coverage of the left subclavian artery (LSA). The LSA was completely covered in patient 1 and patient 6, and partially covered in patient 3 due to a limited landing zone. We chose the left femoral artery as the operative approach in four patients to prevent the impairment of renal function. In two patients whose renal grafts were not perfused, we delivered the stent graft through the right femoral artery. The mean time of operation was 54.2 minutes (48-64 min), and the mean usage of contrast agent was 73.3 ml (60-90 ml).

### Postoperative complications

During postoperative hospitalization, all patients survived without severe complications, including paraplegia, left upper limb ischemia, cardiac or cerebral events and multiple organ failure. While the oxyhemoglobin saturation of patient 3 transiently dropped below 90% on the 3rd day after surgery, the 12th day postoperative CTA showed that the false lumen had already partially thrombosed although pleural effusion was increased. At the 3-month CTA, the pleural effusion disappeared and the false lumen was further narrowed. An increase in pleural effusion was detected in another patient but was absorbed later during follow up. One patient had chest pains after TEVAR that were relieved after 15 days. Patient 2 and patient 4 experienced fever during postoperative hospitalization; this was expected as these two patients received metacortandracin therapy after renal transplantation. The infection was well controlled after antibiotics administration following pharmacy department consultation. Four patients with working renal grafts had mild increase of serum creatinine on 2nd postoperative day; the other two patients received dialysis treatment on 1st postoperative day. Table 1 summarizes the main characteristics and outcomes of the patients.

**Table 1:** Operation related outcomes of the six patients

Variable	Patient 1	Patient 2	Patient 3	Patient 4	Patient 5	Patient 6
Primary tear site	5 mm distal to LSA	25 mm distal to LSA	15 mm distal to LSA	20 mm distal to LSA	35 mm distal to LSA	10 mm distal to LSA
Timing of operation	15 days after onset	10 days after onset	7 days after onset	17 days after onset	22 days after onset	1 year after onset
Type of grafts	Medtronic 34-34-200 mm, Optimed 24-24-80 mm	Life Tech Ankura 28-22-180 mm	Life Tech Ankura 34-28-180 mm	Life Tech Ankura 34-26-180 mm	MicroPort Hercules 34-28-160 mm	Life Tech Ankura 28-22-180 mm
Operative approach	Left femoral artery	Right femoral artery	Left femoral artery	Right femoral artery	Left femoral artery	Right femoral artery
Duration of operation	60 minutes	48 minutes	50 minutes	53 minutes	64 minutes	50 minutes
Volume of contrast agent	60 mL	90 mL	60 mL	90 mL	60 mL	80 mL
Coverage of LSA	Complete	No	Partial	No	No	Complete
Postoperative renal function	Cr 55.20 μmol/L,	Cr 747.40 μmol/L,	Cr 196.0 μmol/L,	Cr 491.80 μmol/L,	Cr 162.50 μmol/L,	Cr 83.70 μmol/L,
	BUN 6.81 mmol/L	BUN 15.23 mmol/L	BUN 7.74 mmol/L	BUN 11.70 mmol/L	BUN 11.10 mmol/L	BUN 7.50 mmol/L
Complications during hospitalization	No	Fever	IPE, Chest pain	IPE, Fever	No	No

Abbreviations: TEVAR = Thoracic Endovascular Aortic Repair; LSA = Left subclavian artery; Cr = Serum creatinine; BUN = Blood urea nitrogen; IPE = Increasing of pleural effusion

Normal range of serum creatinine:44-133μmol/L

Normal range of blood urea nitrogen:3.2-7.1mmol/L

### Follow-up results

Follow-up was done by phone calls and outpatient visits after surgery; the general condition, renal function, blood pressure, and CTA surveillance of the patients were evaluated. CTA was performed before discharge, 3 and 6 months after discharge, and then yearly thereafter. Assessment of endoleak, stent graft migration, and the expansion of aortic diameter was performed by CTA. During the 12-48-month follow-up period, no patients had endoleak or stent graft migration. Thrombosis of the proximal false lumen without enlargement was detected by CTA in all patients, while the retrograde blood flow from distal tear site was present in five patients (Figure 1C-1E). We also found that neither stenosis nor thrombosis of the renal graft artery occurred in four patients, whose renal grafts were functional and perfused preoperatively, while progressive renal graft dysfunction was observed in two patients. The follow-up results showed that serum creatinine levels increased in patient 3 (highest serum creatinine: 357.8 μmol/L). Even worse, patient 5 progressed to renal failure and had hypertension as a result of refusing anti-rejection therapy. Although a 4-year follow-up CTA showed no endoleak or stent graft migration, the patient eventually died of chronic heart failure. The other five patients survived without severe complications during the follow-up period. The postoperative serum creatinine levels in patients during the follow-up period are shown in Figure 2. The follow-up results are summarized in Table 2.

**Figure 1:** Pre-, Intra-, Post-operative imaging of patient 1 **(A)** Aortography showed that the true lumen was compressed at the primary entry tear located at the proximal descending aorta (arrow), 5 mm to the LSA. **(B)** Aortography after stent deployment showed successful endovascular repair of the dissection without endoleak. The bare stent was deployed at the distal descending aorta (arrow). The lumen was expanded by the stent. **(C-E)** The 1st, 6th, 24th month postoperative CTA showed that none of endoleak, malperfusion of renal graft, or stenosis of renal artery was occurred (arrow), but retrograde flow from distal tear site was still existed (triangle).

**Figure 2:** Postoperative serum creatinine levels in TEVAR patients during follow-up period Patient 2 (red) and patient 4 (yellow) had high levels of serum creatinine during the follow-up period, and they needed renal replacement therapy all the time Patient 1 (wathet blue) and patient 6 (green) had normal levels of serum creatinine. The serum creatinine levels of Patient 3 (gray) and Patient 5 (blue) increased during the follow-up period. P, Patient; M, month; Y, year.

**Table 2:** Follow-up results of the six patients

Variable	Patient 1	Patient 2	Patient 3	Patient 4	Patient 5	Patient 6
Follow up duration (months)	31	23	28	30	48	12
Endoleak	No	No	No	No	No	No
Stent-graft migration	No	No	No	No	No	No
Thrombosis of false lumen	Yes	Yes	Yes	Yes	Yes	Yes
Postoperative BP (mmHg)	50-80/100-120	60-90/100-140	65-80/110-130	70-80/100-135	70-100/110-190	60-90/100-130
^*^Renal function	Normal	/	Decreased	/	Decreased	Normal
Current status	Alive	Alive	Alive	Alive	Dead	Alive

Abbreviations: The asterisk (^*^) represents the last observations results during the follow-up period; BP = Blood pressure

## DISCUSSION

The etiology of AD after renal transplantation is multifactorial. Recently, cardiovascular disease (CVD) was reported in 25% to 53% of patients after renal transplantation [13]. Patients with end-stage renal disease (ESRD) carry an increased risk of CVD and acute atherosclerotic vascular events shortly after renal transplantation [14]. Renal stenosis following successful renal transplantation varies from 1% to 25% [15-19]. In our study, we found that there were soft plaques in femoral artery walls during operation in two patients, but there were no obvious calcified plaques on CTA. Renal hypoperfusion occurs in renal artery stenosis, resulting in the activation of the renin-angiotensin-aldosterone system. Patients usually present with worsening or refractory hypertension, fluid retention, and renal graft dysfunction. All our patients were hypertensive; we found that the patients who had renal hypoperfusion were more inclined to have high and unstable BP despite using anti-hypertensive medicine. Preoperative CTA and intraoperative digital subtraction angiography (DSA) showed that the renal grafts of patient 2 and patient 4 were not perfused due to renal artery occlusion (Figure 3A+3C). Compared to the other patients (Figure 3B+3D), they needed stronger anti-hypertension therapy. Thus, the etiology of AD after renal transplantation is multifactorial and complex, and it makes the rupture of AD after renal transplantation unpredictable.

**Figure 3:** Comparison of preoperative CTA results between patient 2 and patient 1 **(A+C)**: Preoperative CTA of patient 2 showed that no perfusion existed in the renal graft of this patient. **(B+D)**: Preoperative CTA of patient 1 showed that the renal graft had normal blood perfusion.

In the past 40 years, we found eleven cases of AD after renal transplantation, including four type A aortic dissections (TAADs) and seven TBADs [20-28]. Robertson reported one case of TBAD after renal transplantation in 1999 [22]; that patient accepted a conservative treatment and was alive during the follow-up period. However, two patients who underwent open surgery died [24, 25]. Only one patient who underwent open surgery survived [26]. Another three patients underwent TEVAR and were alive during the follow up period [27, 28]; one of them needed stenting to cover a re-entry tear site 4 years later after TEVAR [28]. Previous reports have shown that the mortality rate of open surgery could be as high as 66.7%. We believe that TBAD after renal transplantation requires TEVAR instead of conservative treatment or open surgery. In our cohort, all patients were alive except one patient who died of a heart failure 4 years later. Furthermore, the one-year survival rate in our study was 100%. Subsequent follow up showed that no severe complications related to TEVAR occurred in any patient. Whether chronic TBAD should be addressed by TEVAR is still controversial. However, based on our experience, we suggest that either acute or chronic TBAD patients, especially TBAD after renal transplantation, should undergo TEVAR due to the high risk of aortic rupture.

TBAD after renal transplantation should be considered a complicated TBAD because these patients have fragile blood vessels, frequently accompanied by hypertension. In addition, the right iliac artery had been bypassed to the renal artery. Damages may occur to the anastomotic stoma when the stent delivery system goes through the right iliac artery to the aorta, resulting in the impairment of renal function. Fortunately, preoperative CTA showed that the majority of the left iliac artery cavity originated from the true lumen in four patients. Therefore, we chose the left side as the operative approach, and the right side in two patients because of renal graft failure. The stent should be delivered through contralateral side in patients with functional renal grafts. Subsequent CTA showed that no renal artery stenosis or thrombosis was present. Although postoperative follow-up results showed that renal function declined in two patients, we believe that it was related with chronic anti-rejection response, stop using anti-rejection medicine (patient 5), nephrotoxicity of long-term use of medication, and hypoperfusion of renal graft caused by iliac artery dissection. All contrast agents have certain nephrotoxicity, but iodixanol is a non-ionized contrast agent that is characterized by isotonicity and is safer for patients with renal transplantation. Reducing the usage is the key to relieve the renal function damage [28]; adequate hydration and diuresis are helpful for protecting renal function, and dialysis could be adopted if necessary. During the follow-up period, there were no endoleaks, stent migration occurred in all patients. Thrombosis of proximal false lumen was detected in all patients, but distal dissection still existed in five patients. The ratio of true lumen and false lumen (T/F) of proximal thoracic aorta gradually increased in these patients, while the T/F of distal thoracic aorta (on the slice of celiac trunk) was unchanged. Complete repair of AD would eventually be accomplished with the development of new graft and technology; it could not only prevent the rupture of distal dissection, but also reduce the risk of postoperative renal hypoperfusion. Under current technical conditions, processing of proximal tear site is the critical step in the whole operation process. We recommend selecting a stent graft with adequate flexibility and a hydrophilic-coated sheath. Rotation and pushing manipulation should be performed carefully during the passage of the device due to vessel fragility. In addition, in order to redress the sharp angle of the aortic arch and to prevent endoleak or recurrence, the stent graft likely needs a longer proximal landing zone. The LSA of three patients was covered due to an inadequate proximal landing zone, and follow-up results showed that no cerebral hypoperfusion or left upper limb ischemia occurred. The chimney technique or snorkel technique may also be performed in the patients with inadequate proximal landing zones, if necessary.

In conclusion, our study shows that thoracic endovascular repair has satisfying short-midterm results for type B aortic dissection after renal transplantation. Besides, we hold that it need relative longer proximal landing zone for preventing the endoleak and recurrence. However, regular hematodialysis, long-term immunosuppressive therapy, and BP control remain crucial factors to prolong survival. Long-term follow-up studies are needed to evaluate the long-term prognosis of thoracic endovascular repair in these patients.

## MATERIALS AND METHODS

### Patient data

This retrospective study was approved by the Ethics Committee of our hospital, and all patients in the study signed consent forms before the operation. The recruited patients presented with TBAD after renal transplantation and received TEVAR from February 2012 to December 2016. There were five male patients and one female patient aged 29 to 62 years old, with an average age of 42.5 years. The etiology of renal failure was varied: three cases resulted from glomerulonephritis, one case resulted from primary nephritic syndrome, and another two cases were due to acute renal failure. Among them, five cases were acute or subacute AD, and one case was chronic AD. Detailed information regarding these six patients is shown in Table 3.

**Table 3:** Clinical characteristics of patients included in the study

Variable	Patient 1	Patient 2	Patient 3	Patient 4	Patient 5	Patient 6
Gender	Female	Male	Male	Male	Male	Male
Age (years-old)	48	29	32	41	62	43
Etiology of renal failure	CGN	ARF	CGN	NS	CGN	ARF
Time after renal transplantation	6 years	4 years	13 years	8 years	12 years	5 years
The location of renal graft	Right iliac fossa	Right iliac fossa	Right iliac fossa	Right iliac fossa	Right iliac fossa	Right iliac fossa
Anti-rejection medicine	Cyclosporine, Mycophenolate Mofetil, Metacortandracin	Tacrolimus, Metacortandracin	Azathioprine	Tacrolimus, Metacortandracin	Tacrolimus, Azathioprine	Tacrolimus, Mycophenolate, Mofetil
Duration of anti-rejection	6 years	4 years	13 years	8 years	8 years	5 years
Renal function after admission	Cr 51.70 μmol/L, BUN 5.67 mmol/L	Cr 1000.00 μmol/L, BUN 19.23 mmol/L	Cr168.00 μmol/L, BUN 6.29 mmol/L	Cr1107.00 μmol/L, BUN 19.73 mmol/L	Cr 146.90 μmol/L, BUN 13.60 mmol/L	Cr 66.70 μmol/L, BUN 6.60 mmol/L
Co-morbidity	HTN 6 years ^*^: 120/220 mmHg	HTN 4 years ^*^: 110/240 mmHg	HTN 13 years ^*^: 160/220 mmHg	HTN 8 years ^*^: 110/200 mmHg	HTN 14 years ^*^: 110/190 mmHg	HTN 3 years ^*^: 100/200 mmHg
	ATH 2 years					
Symptoms and duration	Chest and back pain, 1 day	Chest and back pain, 11 hours	Chest and back pain, 1 day	Chest and back pain, 10 days	Chest and back pain, 15 days	Mild back pain, 1 year

Abbreviations: CGN = Chronic glomerulonephritis; ARF = Acute renal failure; NS = Nephrotic syndrome; HTN = Hypertension; ATH = Abdominal total hysterectomy; The asterisk (^*^) represents the highest blood pressure.

### TEVAR for aortic dissection

All patients received TEVAR in the catheter room under general anesthesia and endotracheal intubation. After intraoperative angiography, we measured the diameters of the proximal and distal landing zones and selected the appropriate stent grafts that were 10%-20% oversized. We delivered the cover stent graft to the aortic arch through the femoral artery to cover the proximal entry tear with or without coverage of the left subclavian artery. The distal side of the aorta was compressed by the false lumen in patient 1 (Figure 1A), and thus, one bare stent was deployed at the middle segment of the descending aorta before deploying the cover stent graft (Figure 1B). During the procedure, the blood pressure of all patients was maintained between 90/50 mmHg and 110/75 mmHg with intravenous sodium nitroprusside or nitroglycerin to prevent stent graft migration. In addition, in order to minimize damage from the contrast agent (Iodixanol) to renal function, two patients underwent aortography only twice on account of preoperative computed tomography angiography (CTA) showing that their renal arteries were totally occluded (Figure 3A+3C). The other four patients needed abdominal aortography and common iliac arteriography to check the perfusion of their renal grafts. All patients experienced successful delivery and expansion of stent grafts; the primary tear sites were well covered, and proximal blood flow to the false lumen was completely blocked (Figure 1B).

## Abbreviations

AD: aortic dissection
TEVAR: thoracic endovascular repair
TBAD: type B aortic dissection
CTA: computed tomography angiography
VC: vascular calcification
BP: blood pressure
LSA: left subclavian artery
CVD: cardiovascular disease
ESRD: end-stage renal disease
DSA: digital subtraction angiography
TAADs: type A aortic dissections
T/F: The ratio of true lumen and false lumen
